The article "Identification of Ten-Gene Related to Lipid Metabolism for Predicting Overall Survival of Breast Invasive Carcinoma" was published in 2022. Journal: Contrast Media Mol Imaging.

# Identification of Ten-Gene Related to Lipid Metabolism for Predicting Overall Survival of Breast Invasive Carcinoma

**DOI:** 10.1155/2022/8348780

**Published:** 2022-07-11

**Authors:** Zhixing Wang, Fan Wang

**Affiliations:** Medical College, Jiangsu Vocational College of Medicine, YanCheng 224000, Jiangsu, China

## Abstract

**Background:**

Predicting the risk of poor prognosis of breast cancer is crucial to treating breast cancer. This study investigated the prognostic assessment of 10 lipid metabolism-related genes constructed as breast cancer models based on this study.

**Methods:**

The TCGA database was used to obtain clinical information and expression data of breast cancer patients, and GSEA analysis and univariate and multivariate Cox proportional risk regression models were performed to identify lipid metabolism genes closely associated with overall survival (OS) of breast cancer patients and to construct a prognostic risk score model based on lipid metabolism gene markers. The Kaplan–Meier method was used to analyze the survival status of patients with high and low-risk scores, and ROC curves assessed the accuracy of this risk score. Finally, the relationship between this risk score and clinicopathological characteristics of BRCA was analyzed in a stratified manner, and the validity of this risk score as an independent prognostic factor was determined using univariate and multivariate Cox regression analyses.

**Results:**

One hundred and forty-four differentially expressed lipid metabolism-related genes were identified in cancer and paracancerous tissues in BRCA, 21 of which were associated with overall survival (OS) in BRCA (*P* < 0.05). Univariate and multivariate Cox analyses revealed that age, grade, and risk score were independent prognostic factors for BRCA. Multivariate Cox regression analysis further identified APOL4, NR1H3, SLC25A5, APOL3, OSBPL1A, DYNLT1, IMMT, MAP2K6, ZDHHC8, and RAB2A lipid metabolism-related genes as independent prognostic markers for BRCA. A prognostic risk score model was developed by labeling lipid metabolism genes with these 10 genes, and patients with BRCA with high-risk scores in the model sample had significantly worse OS than those with low-risk (*P* < 0.01). The ROC curve area (AUC) of this risk score model was 0.712.

**Conclusion:**

By mining the TCGA database, we identified 10 lipid metabolism-related genes APOL4, NR1H3, SLC25A5, APOL3, OSBPL1A, DYNLT1, IMMT, MAP2K6, ZDHHC8, and RAB2A, which are closely related to the prognosis of BRCA patients, and constructed a prognostic risk scoring system based on 10 lipid metabolism genes tags.

## 1. Background

According to statistics, in 2020, for the first time, breast cancer in women will overtake lung cancer as the most common cancer worldwide [1]. Currently, the main treatments for breast cancer include surgery, chemotherapy, radiotherapy, and targeted therapy, but all have varying degrees of side effects that affect the prognosis of patients [1]. Therefore, predicting the risk of poor prognosis in breast cancer is crucial for breast cancer treatment. Lipids are widely distributed in cellular organelles and are a crucial part of all membranes; they form the basic structure of membranes, signal molecules, and energy sources [2, 3]. There is growing evidence that the lipid metabolism is largely reprogrammed in cancer [4, 5] and that lipid production in human cancers is strongly upregulated to meet the demands of increased membrane biogenesis [6, 7]. Most types of cancers use lipids and cholesterol to meet their unlimited energy requirements [8]. Increased lipid uptake, storage, and lipogenesis have been shown to occur in various cancers and contribute to rapid tumor growth [9]. Based on this background, this study used the TCGA database to obtain clinical information and expression data of breast cancer patients, identified lipid metabolism genes that are closely associated with overall survival (OS) of breast cancer patients, and constructed a prognostic risk scoring system based on 10 lipid metabolism gene tags, which provides new targets for diagnosis and treatment of breast cancer and can promote human understanding of the pathogenesis of breast cancer and improve. It can promote human understanding of the pathogenesis of breast cancer and improve diagnosis and treatment.

## 2. Methods

### 2.1. Collection of Genetic and Clinical Data

Breast cancer patients' clinical data and mRNA expression profiles were downloaded from the TCGA database (https://portal.gdc.cancer.gov/). The selection criteria were set as the primary cancer site was the breast, the project name was TCGA-BRCA, the expression data type was HTSeq–FPKM, the data type was a transcript, and the experimental method was RNA-Seq technology. This data matrix contains 1109 breast cancer patients and 113 healthy controls. The dataset of 8 genes related to the lipid metabolism was downloaded from the GSEA official website (https://www.gsea-msigdb.org/gsea/downloads.jsp).

### 2.2. Gene Set Enrichment Analysis

The eight downloaded datasets were enriched and analyzed with GSEA 4.1.0, and validated lipid metabolism-related gene datasets with standardized *P* < 0.05 were screened separately. Lipid metabolism genes and their expressions were extracted from these 8 datasets, screened for *P* < 0.05 differential analysis using the limma package, and combined the differential gene expression and survival data.

### 2.3. Construction of a Prognostic Model for Lipid Metabolism

Univariate Cox regression analysis was applied to identify lipid metabolism-related genes associated with overall survival, and then, multivariate Cox regression was performed to screen out the prognosis-related lipid metabolism genes and obtain the hazard ratio (HR). The screened lipid metabolism genes were then classified into hazard (HR > 1) and protective (0 < HR < 1) types. A prognostic risk score model was constructed according to the linear combination of expression levels, and the regression coefficients obtained by multivariate Cox regression analysis were weighted with the following risk parameter formula: risk parameter = ∑ (*βn* × expression of gene *n*).

Using the survival package in R 4.0.2, a prognostic model of the lipid metabolism in breast cancer with minimal AIC value was constructed by multifactorial COX regression, and the risk values of patients were output. The survival curves of the 2 groups were plotted according to the median value divided into 2 groups of high and low risks, and the risk curves were plotted using ROC curves to judge the validity of the model diagnosis.

### 2.4. Lipid Metabolism-Related Features Are Independent Prognostic Factors for Breast Cancer

Univariate and multivariate Cox regression analyses and data stratification analyses were performed to assess whether risk scores were independent of clinical characteristics. *P* < 0.05 was considered statistically significant.

#### 2.4.1. Mutation and Difference Analysis of Model Gene

Mutations in model genes were analyzed using the online network (https://www.cbioportal.org/), and breast cancer samples were selected from the TCGA dataset to analyze the frequency and type of mutations in lipid metabolism genes of tumors in the prognostic model. All steps were performed according to the cBioPortal instructions.

### 2.5. Statistical Analysis

Using Kaplan–Meier survival curves and the log-rank method (Log-rank), the accuracy of risk parameters was estimated. Multivariate Cox analyses were then performed to test whether risk parameters were independent of other clinical characteristics, and all statistical analyses were performed using R 4.0.2, with *p* < 0.05 being statistically significant.

## 3. Results

### 3.1. Enrichment Analysis of Lipid Metabolism in Thyroid Carcinoma

The clinical data and mRNA expression datasets of 1109 BRCA patients were obtained from The Cancer Genome Atlas (TCGA). After screening 8 datasets, 5 datasets were finally found to be eligible, and GSEA analysis of 1494 genes involved in lipid metabolic processes revealed that most of these genes were more active in the tumor samples. Values (*P*), where FDR < 0.1 and *P* < 0.05, were used to screen eligible gene sets, and FDR was performed for lipid metabolism gene subset size and multiple hypothesis test correction (Figure 1). GSEA determined that KEGG_ARACHIDONIC_ACID_METABOLISM, KEGG_ETHER_LIPID_METABOLISM, KEGG_GLYCEROLIPID_METABOLISM, KEGG_GLYCEROPHOSPHOLIPID_METABOLISM, and WP_LIPID_METABOLISM_PATHWAY are five sets of lipid metabolism-related genes upregulated in BRCA.

### 3.2. Lipid Metabolism Genes Related to the Prognosis of Thyroid Carcinoma

Univariate Cox regression analysis was performed on the expression of lipid metabolism-related genes in eight genomes in BRCA to identify prognostically relevant differentially expressed genes for the lipid metabolism. The data showed that the expression of 21 differentially expressed lipid metabolism-related genes was associated with OS in patients with BRCA (*P* < 0.05) (Table 1). Next, multivariate Cox regression analysis was performed to identify further 10 lipid metabolism-related genes APOL4, NR1H3, SLC25A5, APOL3, OSBPL1A, DYNLT1, IMMT, MAP2K6, ZDHHC8, and RAB2A as independent prognostic markers for BRCA, with SLC25A5, DYNLT1, and HRs for IMMT and RAB2A identified. With HRs greater than 1 for IMMT and RAB2A, risk phenotypes are with low patient survival (Table 2).

### 3.3. Prognostic Model of Lipid Metabolism in Thyroid Carcinoma

A prognostic model consisting of APOL4, NR1H3, SLC25A5, APOL3, OSBPL1A, DYNLT1, IMMT, MAP2K6, ZDHHC8, and RAB2A was constructed by multifactorial COX regression based on the risk value = APOL4 expression × 0.9478 + NR1H3 expression × 0.9531 + SLC25A5 expression × 1.0018 ＋ APOL3 expression × 0.9698 ＋ OSBPL1A expression × 0.9553 ＋ DYNLT1 expression × 1.0107 ＋ IMMT expression × 1.0181 ＋ MAP2K6 expression × 0.7772 ＋ ZDHHC8 expression × 0.9454 ＋ RAB2A expression × 1.0093 and the value was calculated. According to their median, the patients were then divided into 2 groups of high and low risks, with 545 breast cancer samples in the high-risk group and 545 breast cancer samples in the low-risk group. The prognosis of the high and low-risk groups was significantly different (*P* < 0.01), as shown by the survival curves (Figure 2(a)). The ROC curve showed that the AUC value was 0.712, indicating the model's predictive value (Figure 2(b)).

### 3.4. Risk Curve

Risk parameters were calculated for each patient, and the patients were divided into high and low-risk groups using the median. The distribution of patients' risk scores (Figure 3(a)) and survival status (Figure 3(b)) are shown. In addition, the heat map shows the expression of the 10 mRNAs (Figure 3(c)). As patients' risk scores increased, the proportion of patients who died gradually increased, and the survival time was significantly shortened. Meanwhile, SLC25A5, DYNLT1, IMMT, and RAB2A were highly expressed in the high-risk group.

### 3.5. Independent Prognostic Analysis of Univariate and Multivariate

Comparing the prognostic value of risk parameters with clinicopathological parameters by univariate and multifactorial analyses showed that gender was not a good predictor of prognosis in breast cancer patients. In contrast, the prognostic model studied here, age, grading, and risk score, could effectively assess the prognosis of patients with a *p* value less than 0.01, showing a significant prognostic value (Figure 4).

### 3.6. Mutation and Difference Analysis of Model Gene

Alterations in 10 risk genes were evaluated by analyzing 996 BRCA samples from the cBioPortal database (https://cbioportal.org). The APOL4 gene was altered in 0.4% of cases, showing amplification mutations and deep deletions. NR1H3 gene was altered in 0.8% of cases, showing amplification mutations, deep deletions, and missense mutations. The SLC25A5 gene was altered in 0.5% of cases, showing amplification mutations and deep deletions. APOL3 gene was altered in 0.6% of cases, showing amplification mutations, deep deletions, and missense mutations. The DYNLT1 gene was altered in 1.2% of cases, showing amplification mutations and deep deletions. The IMMT gene was altered in 0.9% of cases, showing amplification mutations, deep deletions, truncation, and missense mutations. The ZDHHC8 gene was altered in 1.2% of cases with amplification mutations, deep deletions, truncation mutations, and missense mutations, and the MAP2K6 and RAB2A genes were altered in 6% of cases with amplification mutations and missense mutations (Figure 5).

The expression of APOL4, NR1H3, SLC25A5, APOL3, OSBPL1A, DYNLT1, IMMT, MAP2K6, ZDHHC8, and RAB2A was upregulated in both normal and tumor samples. *P* value for APOL3, MAP2K6, RAB2A, and ZDHHC8 was less than 0.05, a significant difference; DYNLT1, IMMT, NR1H3, OSBPL1A, and SLC25A5 had a *P* value less than 0.001, and the difference was highly significant (Figure 6).

### 3.7. Model Validation of Survival Curves for Clinical Characteristics and Clinical Subgroups

Both univariate and multivariate Cox regression analyses of OS revealed several clinicopathological parameters that predict BRCA survival, including age, grade, and risk score. We then validated these findings using Kaplan–Meier survival curves, which showed consistent results with age (Figure 7(a)), stage (Figure 7(c)), T-stage (Figure 7(d)), N-stage (Figure 7(e)), and M-stage (Figure 7(f)) being associated with poor prognosis. These results further confirm the reliability of the analysis.

Several clinical characteristics were evaluated by Kaplan–Meier analysis using log-rank tests to assess the predictive ability of BC patients. The results showed that the survival curve was not affected by the age >65 group (Figure 8(a)), and the prognosis of patients in the male subgroup with high-risk scores was not significant and could not be used to predict the prognosis of patients with BRCA (Figures 8(c) and 8(d)). However, when we divided BRCA patients into different subgroups according to TNM, the risk parameter could no longer be used as the M1 subgroup alone (Figure 8(l)), suggesting that this risk parameter is influenced by TNM staging BRCA patients, which needs to be further explored.

## 4. Conclusions

This study focused on assessing the prognosis of breast cancer by a model constructed from genes related to the lipid metabolism. It was shown that univariate and multifactorial Cox analyses showed that age, grade, and risk score were independent prognostic factors for BRCA, and the study was statistically significant. The results showed that DYNLT1, IMMT, RAB2A, and SLC25A5 were unfavorable factors for breast cancer prognosis in the lipid metabolic pathway. APOL3, APOL4, NR1H3, OSBPL1A, MAP2K6, and ZDHHC8 were protective genes for breast cancer prognosis.

It is well known that APOL3-controlled NCS-1 promotes cancer cell motility, metastatic spread, and survival. The reduction of *π* (4) *P* observed in human breast cancer, where Golgi *π* (4) *P* is a regulator of cell adhesion and invasive cell migration [10, 11]. APOL1Δ and APOL3KO foot cells can be responsible for this metastatic phenotype. APOLs are suspected to be involved in various cancers, including cervical, ovarian, breast, thyroid, bladder, prostate, and colorectal cancers [12–15]. It is known that NR1H3 is involved in various metabolic functions such as cholesterol, fatty acid and glucose homeostasis, and steroidogenesis. The main physiological functions of NR1H3 are maintenance of cholesterol levels, lipoprotein metabolism, and lipid synthesis, and at high cholesterol levels, NR1H3 is a major transcriptional regulator involved in lipid metabolism gene synthesis [16–18]. Oxygen sterol binding protein-related protein 1 (OSBPL1A) is an intracellular lipid receptor and a member of the oxygen sterol binding protein (OSBP) family [19]. The familial loss-of-function mutation in OSBPL1A affects the first step of the reverse cholesterol transport process and is associated with a low HDL-C phenotype, suggesting that rare mutations in the OSBPL gene may contribute to dyslipidemia [20]. MAP2K6 is involved in various physiological and pathological processes, such as cell growth, development, division, and inflammatory responses. In recent years, it has been found that MAP2K6 may be associated with tumorigenesis and progression [21]. MAP2K6 may be involved in human tumorigenesis and progression and may be considered a new diagnostic or prognostic biomarker for cancer [22, 23]. Previous studies have shown that MAP2K6 plays a vital role in cell cycle regulation, transcription, and apoptosis. Parray et al. [15] found significantly higher expression of MAP2K6 in esophageal, gastric, and colon cancers than in controls using protein blotting and immunofluorescence assays, and overexpression of MAP2K6 suggests a role in human cancers. It may be a novel diagnostic or prognostic biomarker in these cancers [24–28]. DHHC8 is localized in mitochondria and is involved in mitochondrial-regulated apoptosis [29]. DYNLT1 is an integral 14 KDa protein subunit of the large microtubule-based cytoplasmic dynein complex [30]. Wei et al. [31] hypothesized that DYNLT1 is associated with apoptosis regulation [31]. In addition, DYNLT1 was previously considered an interaction partner of REIC/Dkk-3, inducing apoptosis through its role as a tumor suppressor in various cancer cell lines [32]. IMMT is a mitochondrial protein that affects the morphological structure and has a putative impact on mitochondrial function. Although there is little knowledge about the function of IMMT, alterations in this marker have been reported in association with different diseases, including Down syndrome, diabetic cardiomyopathy, and Parkinson's disease [33–37].

This study constructs a prognostic risk score model based on lipid metabolism gene labeling and validates it by survival analysis, ROC curve plotting, risk function assessment, and independent prognostic analysis. We found that DYNLT1, IMMT, RAB2A, and SLC25A5 were tumor biomarkers to assess the prognosis of BRCA patients, and all of them were high-risk genes, and the parameters indicated that 4 genes would make the prognosis of BRCA poorer. These results provide new ideas and approaches for developing drugs targeting the energy metabolism of BRCA cells and for the clinical treatment of BRCA.

## Figures and Tables

**Figure 1:** Enrichment analysis of lipid metabolism gene set. (a) *P* = 0.003, KEGG_ARACHIDONIC_ACID_METABOLISM. (b) *P* = 0.005, KEGG_ETHER_LIPID_METABOLISM. (c) *P* = 0.021, KEGG_GLYCEROLIPID_METABOLISM. (d) *P* = 0.037, KEGG_GLYCEROPHOSPHOLIPID_METABOLISM. (e) *P* = 0.013, WP_LIPID_METABOLISM_PATHWAY.

**Figure 2:** Survival analysis of the lipid metabolism prognostic model with ROC curves.

**Figure 3:** Risk curve.

**Figure 4:** Independent prognostic analysis.

**Figure 5:** Mutations in prognostic model genes.

**Figure 6:** Differential analysis of prognostic model genes.

**Figure 7:** Relationship between risk score distribution and clinical parameters.

**Figure 8:** Kaplan–Meier curves to assess the prognostic value of risk parameters in patients grouped by clinical characteristics.

**Table 1:** 21 univariate Cox regression-associated lipid metabolism genes in breast cancer.

Gene	HR	HR.95L	HR.95H	Cox *P* value
APOL4	0.900877879	0.834348061	0.972712697	0.00765844
NR1H3	0.919241179	0.865931412	0.975832881	0.005735271
SLC25A5	1.001960965	1.000317045	1.003607587	0.019370037
APOL3	0.948868181	0.913186198	0.985944408	0.007279521
OSBPL1A	0.959529209	0.923596388	0.996860007	0.03388302
DYNLT1	1.017520083	1.005999394	1.029172708	0.002794158
HSPA9	1.009104615	1.004457297	1.013773434	0.000118927
SLC35A2	1.025997849	1.009627085	1.042634059	0.001763323
ENPP6	0.400790856	0.165340628	0.971529573	0.042980469
IMMT	1.021791143	1.00438895	1.03949485	0.013907542
GBP2	0.980967649	0.967334692	0.994792739	0.007120906
MAP2K6	0.767586959	0.616910246	0.955065576	0.017677113
ZDHHC8	0.910449729	0.845440542	0.980457723	0.013060524
HSPA4	1.010302771	1.001638957	1.019041523	0.019666949
KDELR2	1.005368525	1.001401791	1.009350973	0.007943869
YWHAB	1.005431653	1.002346635	1.008526165	0.000550569
DENND5A	0.948306241	0.899822755	0.999402073	0.047445508
RAB2A	1.01409836	1.00636175	1.021894447	0.000339738
WLS	0.980395937	0.962721035	0.998395337	0.032926553
KDELR1	1.003917855	1.000416053	1.007431914	0.028286843
ZDHHC9	1.032053594	1.012770657	1.051703674	0.001043034

**Table 2:** 10 multivariate Cox regression-associated lipid metabolism genes in breast cancer.

Id	Coefficient	HR
APOL4	−0.053646743	0.947766852
NR1H3	−0.048036694	0.953098814
SLC25A5	0.001753325	1.001754863
APOL3	−0.030663112	0.969802232
OSBPL1A	−0.045680466	0.95534718
DYNLT1	0.010606609	1.010663058
IMMT	0.017937573	1.018099418
MAP2K6	−0.252082595	0.777180544
ZDHHC8	−0.056161117	0.945386806
RAB2A	0.009273916	1.009317052

## Data Availability

The datasets generated during this study are available in the TCGA database (https://portal.gdc.cancer.gov/repository).

## Abbreviations

abrBRCA: Breast invasive carcinoma
TCGA: The Cancer Genome Atlas
GSEA: Gene set enrichment analysis
GSVA: Gene set variation analysis
GO: Gene ontology
KEGG: Kyoto Encyclopedia of Genes and Genomes
WGCNA: Weighted correlation network analysis
ROC: Receiver operating characteristic
AUC: Area under the ROC curve
TME: Tumor microenvironment
TNM: Tumor-node-metastasis
FC: Fold change.
